# Standardization of Environmental Responsibility Behavior of Production and Manufacturing Enterprises in the Context of Green Economy

**DOI:** 10.1155/2022/2746263

**Published:** 2022-08-10

**Authors:** Lei Chen, Wen Lin

**Affiliations:** School of Accountancy, Wuhan Textile University, Wuhan 430200, China

## Abstract

The motivation and decision-making of an enterprise are significantly affected by the green economy and the environmental and economic policies (EEPs). It is practical to deeply analyze the standardization mechanism and actual effect of environmental responsibility behavior (ERB) in enterprises. This study explores the ERB standardization in the context of green economy. First, a conceptual model was established for the action mechanism of the factors driving ERB standardization in enterprises, and an empirical model was developed around the concept of policy-behavior-performance, before investigating the influence of the ERB of production and manufacturing enterprises (PMEs) over their production benefit (PB). From the angle of motivation-supervision theory, the authors examined how the supervision and motivation of EEPs affect the large panel PMEs' sense of social responsibility (SSR) and ERB. Finally, the variables like marketization index (MI) and return on assets (ROA) were regressed, and the ERB standard level of PMEs in different industries was analyzed statistically. The results demonstrate the robustness of our empirical model. Finally, opinions and suggestions were provided to guide or constrain environmental and economic policies.

## 1. Introduction

The traditional long-term extensive model of economic development has also brought tremendous pressure on China's natural environment [1–3] and constrains the economic transformation from low-speed development and high-speed development to high-quality development [4–7]. As the main body of socioeconomic activities and pollution emissions, production and manufacturing enterprises (PMEs) play an important role in promoting the progress of socioeconomic development, the innovation and application of science and technology, and the production and allocation of natural resources [8–13]. During the pursuit of the maximal interests, the enterprises inevitably pollute the natural environment, and they must shoulder the social responsibility of governing the environmental pollution [14–18]. The motivation and decision-making of an enterprise are significantly affected by the green economy and the environmental and economic policies (EEPs) [19, 20]. It is practical to deeply analyze the standardization mechanism and actual effect of environmental responsibility behavior (ERB) in enterprises. The analysis could provide a theoretical support in solving the existing problems.

Green innovation and pollutant emissions are the hottest topics in the current research of ERB among enterprises. Peng et al. [21] adopted the multinomial Logit model to discuss the internal selection logic of the Chief Executives Board for Coordination. The model considers the choices of green innovation and illegal emissions made by enterprises in different regions of China. Focusing on the duopoly market, Pu and Tian [22] constructed the Stackelberg game model for the leading manufacturing enterprise and the following manufacturer enterprise and systematically analyzed the influence of subsidy policies on low-carbon production behavior.

In the game of environmental governance, the strategic choices of the government and enterprises determine the effect of environmental governance. Tian [23] established an asymmetric evolution game model between the government and enterprises. The stability theorem of differential equations was drawn to discuss the strategic evolution path of each player and identify the factors affecting the evolution. In addition, the evolutionarily stable strategy (ESS) of the game system was determined with the Jacobian matrix.

Enterprises regard environmental protection as a constraint on their economic activities because it slowly lower the profitability and competitiveness by limiting the freedom of production and response and bringing an additional cost to meet environmental regulations. Pang and Xiaolei [24] introduced the definition, classification, channels of environmental regulations, and corporate behavior. Then, the influence of environmental regulation on corporate behavior was discussed, including profit maximization, technological innovation, and competitive behavior.

Reducing innovation cost and providing innovation subsidy can stimulate private enterprises to transform their production model to green production. Based on the computing experimental method in social sciences, Guan et al. [25] built a dynamic model of the environmental innovation behavior of private enterprises, simulated the evolution of private enterprises under different market mechanisms, product competition, and innovation subsidy, and examined the influence of different subsidy models on the innovation of environmental technologies.

On the ERB standardization of PMEs in the context of green economy, many theoretical and empirical results have been achieved. But most of the results belong to the macroscale. In addition, the ideal effect cannot be achieved with the existing standards of data collection, utilization, and measurement and the current measuring methods. Therefore, this study further explores the ERB standardization of PMEs in the context of green economy.

The variables like marketization index (MI) and return on assets (ROA) were regressed, and the ERB standard level of PMEs in different industries was analyzed statistically. The results showed that the mean and median of the PMEs under EEP regulation were not different. This means most enterprises differ slightly in the marketization level. But very few enterprises diverge significantly in that respect.

## 2. Empirical Model

As judged by the ERB, implemented by Chinese PMEs, the EEPs in the context of green economy are the main influencing factors of corporate ERB.  Figure 1 shows the conceptual model for the action mechanism of the factors driving ERB standardization in enterprises. These drivers contain external factors and internal factors. The external factors include EEP constraint, ERB standard, and market effect, while the internal factors include subjective cognition and SSR. These factors mainly belong to three aspects of corporate ERB: speculation behavior control, green production, and green process innovation.

After combing through the relevant literature, it was learned that the implementation of ERB is mainly motivated by the EEP regulation of the government and the concentration of the local industry and not greatly affected by the social and cultural values. Hence, our analysis unfolds from the angles of EEP regulation and industry concentration. During the development, PMEs always pursuit the maximal PB. To disclose the influence of PMEs' ERB on their PB, this study develops an empirical model around the concept of policy-behavior-performance.

The correlation between EEP regulation and PMEs' ERB can be tested by the following regression model:

(1) $$\begin{array}{c} \text{HTQ}=\beta +\gamma_{1}\text{MAR}+\gamma_{2}\text{ADU}+\gamma_{3}\text{HR}+\gamma_{4}\text{CD}+\gamma_{5}\text{GV}+\gamma_{6}\text{TJ}+\gamma_{7}\text{EC}+\gamma_{8}\text{EQ}+\gamma_{9}\text{WE}+\gamma_{10}\text{DE}+\gamma_{11}\text{MEU}+\sigma , \end{array}$$

where *β* is a constant term, *γ*_*i*_ (*i* = 1,2,3,…, 11) are the coefficients, *σ* is a random error, MAR is the MI, HTQ is the environmental investment intensity, ADU is the asset-liability ratio, HR is the growth rate of operating income, CD is the enterprise scale, GV is the surviving time of the enterprise, TJ is the investment opportunity, EC is the equity concentration, EQ is the degree of balance of shareholder power, WE is the proportion of independent directors, MEU is the return on investment, and DE is whether the chairman also serves as the general manager. The given random error (*σ*) is assumed to be normally distributed with zero mean value and constant variance [26, 27].

Let FGT denote the industry concentration of the enterprise. Then, the correlation between industry concentration and PMEs' ERB can be tested by the following regression model:

(2) $$\begin{array}{c} \text{HTQ}=\beta +\gamma_{1}\text{FGT}+\gamma_{2}\text{ADU}+\gamma_{3}\text{HR}+\gamma_{4}\text{CD}+\gamma_{5}\text{GV}+\gamma_{6}\text{TJ}+\gamma_{7}\text{EC}+\gamma_{8}\text{EQ}+\gamma_{9}\text{WE}+\gamma_{10}\text{DE}+\gamma_{11}\text{MEU}+\sigma . \end{array}$$

The form of PME ownership regulates the relationship between EEP regulation and PMEs' ERB. The regulating effect can be characterized by the cross-term between the independent variable and the moderator variable. Let FEO denote the form of PME ownership. Then, the following regression model can be established:

(3) $$\begin{array}{c} \text{HTQ}=\beta +\gamma_{1}\text{MAR}+\gamma_{2}\text{FEO}+\gamma_{3}\text{MAR}*\text{FEO}+\gamma_{4}\text{ADU}+\gamma_{5}\text{HR}+\gamma_{6}\text{CD}+\gamma_{7}\text{GV}+\gamma_{8}\text{TJ}+\gamma_{9}\text{EC}+\gamma_{10}\text{EQ}+\gamma_{11}\text{WE}+\gamma_{12}\text{DE}++\gamma_{13}\text{MEU}+\sigma . \end{array}$$

The regulating effect of FEO on the relationship between industry concentration and PMEs' ERB can be tested by the following regression model:

(4) $$\begin{array}{c} \text{HBG}=\beta +\gamma_{1}\text{FGT}+\gamma_{2}\text{FEO}+\gamma_{3}\text{FGT}*\text{FEO}+\gamma_{4}\text{ADU}+\gamma_{5}\text{HR}+\gamma_{6}\text{CD}+\gamma_{7}\text{GV}+\gamma_{8}\text{TJ}+\gamma_{9}\text{EC}+\gamma_{10}\text{EQ}+\gamma_{11}\text{WE}+\gamma_{12}\text{DE}++\gamma_{13}\text{MEU}+\sigma . \end{array}$$

Let ZBL denote the ROA of the enterprise. The correlation between PMEs' ERB and its PB can be tested by the following regression model:

(5) $$\begin{array}{c} {\text{ZBL}}_{o}=\beta +\gamma_{1}\text{HTQ}+\gamma_{2}\text{ADU}+\gamma_{3}\text{HR}+\gamma_{4}\text{CD}+\gamma_{5}\text{GV}+\gamma_{6}\text{TJ}+\gamma_{7}\text{EC}+\gamma_{8}\text{EQ}+\gamma_{9}\text{WE}+\gamma_{10}\text{DE}+\gamma_{11}\text{MEU}+\sigma . \end{array}$$

## 3. ERB Standardization Model

Our research intends to answer the following questions: How does the supervision and motivation mechanism of government departments affect the ERB of enterprises? How does the SSR of enterprises influence the standardization of their ERB? To this end, an empirical model was developed around the concept of policy-behavior-performance and used to investigate the influence of government measures of supervision and motivation over the ERB of enterprises.

For a long time, large panel PMEs are not fully aware of the innovation and development of green production processes. With the rising production costs and limited income, the PMEs lack the motivation to implement green production.

Despite that, the society now attaches a great importance to greenness and environmental protection. Since the conceptualization of green economy, PMEs could acquire more financial subsidy and preference for green production, particularly as the government rolls out EEPs and the regulatory departments step up supervision. Against this backdrop, PMEs are increasingly aware of the importance of innovating and developing green production processes.

Figure 2 shows the driving mechanism of large panel PMEs' ERB. It can be seen that the standardization conditions and environmental policies, coupled with SSR, drive PMEs to optimize their production structures and implement mature ERB.

The level of government motivation is the main factor affecting the contract execution of large panel production enterprises, while the supervision and penalty intensity of the government do not affect their contract execution. From the angle of motivation-supervision theory, the authors examined how the supervision and motivation of EEPs affect the large panel PMEs' SSR and ERB.

The behavior of large panel PMEs can be divided into the behavior that benefits green production *φ*_*h*_ and the opportunistic behavior *φ*_*y*_. The costs of *φ*_*h*_ and *φ*_*y*_ are denoted by *d*(*φ*_*h*_) and *d*(*φ*_*y*_), respectively. The two costs satisfy *d*'(*φ*_*h*_) > 0, *d*(*φ*_*h*_) > 0, and *d*'(*φ*_*y*_) > 0, *d*(*φ*_*y*_) > 0. The functions of *d*(*φ*_*h*_) and *d*(*φ*_*y*_) can be expressed as *d*(*φ*_*h*_) = *y*_*h*_*φ*_*h*_^2^/2 and *d*(*φ*_*y*_) = *y*_*y*_*φ*_*y*_^2^/2, respectively.

The benefit of large panel PMEs is the joint result of green production and opportunistic behavior of enterprises: Ψ = *φ*_*h*_−*φ*_*y*_ + *ω*, where *ω* obeys the *N*(0, *ε*^2^_1_) distribution. On this basis, it is assumed that the influence of EEP constraint on PMEs is *l*(0 ≤ *l* ≤ 1). The probability of being constrained by EPPs is denoted as *d*(*l*) > 0 and the corresponding EEP constraint cost as *d*(*l*). The condition meeting *d'*(*l*) > 0 can be described by the function *d*(*l*) = *Nl*^2^/2, where *N* is the cost coefficient.

Under the constraint of EEPs, any PME failing to implement the environmental responsibility, i.e., committing opportunistic behavior, will be penalized. The penalty coefficient *G* satisfies *G*(*φ*_*y*_) = *Gφ*_*y*_, that is, the penalty increases with the severity of the opportunistic behavior. The EEP constraint intensity and penalty intensity are denoted by *lG*(*φ*_*y*_) = *lGφ*_*y*_ and *lG*, respectively.

The income of PMEs comes from two sources: the sum *r*_1_ of the normal production income and the financial subsidy and preference for green production; the gray income *r*_2_ of committing opportunistic behavior. The two parts *r*_1_ and *r*_2_ of income are independent of each other. Thus, the covariance of the two can be regarded as zero. Specifically, *r*_1_ and *r*_2_ can be expressed as *r*_1_ = *θ* + *απ* = *θ* + *α*(*φ*_*h*_ − *φ*_*y*_ + *ω*), with 0 < *α* *≤* 1, and *r*_2_ = *Kφ*_*y*_ + *σ*, with *σ* obeying the *N*(0, *ε*^2^_2_) distribution, respectively. Then, the total income of a PME can be expressed as *r* = *r*_1_ + *r*_2_ = *θ*+*α*(*φ*_*h*_−*φ*_*y*_ + *ω*) + (*Kφ*_*y*_ + *σ*). Finally, the reservation utility of PMEs is denoted as *θ*.

On this basis, the expected income under the constraint of EEPs can be calculated by

(6) $$\begin{array}{c} Q^{T}=Q\left(\Psi -r_{1}-d\left(l\right)+lG\phi_{y}\right)=\left(1-\alpha \right)\left(\phi_{h}-\phi_{y}\right)-\theta -\frac{NL^{2}}{2}+lG\phi_{y}. \end{array}$$

The actual profit of large panel PMEs can be calculated by

(7) $$\begin{array}{c} Q^{X}=Q\left(r_{1}+r_{2}-d\left(\phi_{h}\right)-d\left(\phi_{y}\right)-LG\phi_{y}\right)=\theta +\alpha \left(\phi_{h}-\phi_{y}\right)+K\phi_{y}-\frac{y_{h}\phi_{h}^{2}}{2}-\frac{y_{y}\phi_{y}^{2}}{2}-lG\phi_{y}. \end{array}$$

The enterprise utility can be characterized by the certain equivalized disposable income as

(8) $$\begin{array}{c} DQ^{X}=\theta +\alpha \left(\phi_{h}-\phi_{y}\right)+K\phi_{y}-\frac{y_{h}\phi_{h}^{2}}{2}-\frac{y_{y}\phi_{y}^{2}}{2}-lG\phi_{y}-\frac{1}{2}\tau \left(\alpha^{2}\varepsilon_{1}^{2}+\varepsilon_{2}^{2}\right). \end{array}$$

The corresponding constraints can be expressed as

(9) $$\begin{array}{c} \left(IS\right)\theta +\alpha \left(\phi_{h}-\phi_{y}\right)+K\phi_{y}-\frac{y_{h}\phi_{h}^{2}}{2}-\frac{y_{y}\phi_{y}^{2}}{2}-lG\phi_{y}-\frac{1}{2}\tau \left(\alpha^{2}\varepsilon_{1}^{2}+\varepsilon_{2}^{2}\right)\geq \Psi . \end{array}$$

The constraints of financial subsidy and preference can be expressed as

(10) $$\begin{array}{c} \left(I\;D\right)\underset{\phi_{h},\phi_{y}}{\max}+\alpha \left(\phi_{h}-\phi_{y}\right)+K\phi_{y}-\frac{y_{h}\phi_{h}^{2}}{2}-\frac{y_{y}\phi_{y}^{2}}{2}-lG\phi_{y}-\frac{1}{2}\tau \left(\alpha^{2}\varepsilon_{1}^{2}+\varepsilon_{2}^{2}\right). \end{array}$$

Through the above analysis, the following game model can be established:

(11) $$\begin{array}{c} \underset{\phi_{h},\phi_{y}}{\max}\left(1-\alpha \right)\left(\phi_{h}-\phi_{y}\right)-\theta -\frac{Nl^{2}}{2}+lG\phi_{y}, \end{array}$$

(12) $$\begin{array}{c} \left(IS\right)\theta +\alpha \left(\phi_{h}-\phi_{y}\right)+K\phi_{y}-\frac{y_{h}\phi_{h}^{2}}{2}-\frac{y_{y}\phi_{y}^{2}}{2}-lG\phi_{y}-\frac{1}{2}\tau \left(\alpha^{2}\varepsilon_{1}^{2}+\varepsilon_{2}^{2}\right)\geq \mathrm{\Psi ,} \end{array}$$

(13) $$\begin{array}{c} \left(I\;D\right)\underset{\phi_{h},\phi_{y}}{\max}\omega +\alpha \left(\phi_{h}-\phi_{y}\right)+K\phi_{y}-\frac{y_{h}\phi_{h}^{2}}{2}-\frac{y_{y}\phi_{y}^{2}}{2}-lG\phi_{y}-\frac{1}{2}\tau \left(\alpha^{2}\varepsilon_{1}^{2}+\varepsilon_{2}^{2}\right). \end{array}$$

## 4. Experiments and Results Analysis

Table 1 provides the descriptive statistics of the main variables in the empirical model based on the concept of policy-behavior-performance. It can be seen that the mean of PMEs implementing ERB was greater than the median. Thus, the enterprises emitting lots of industrial solid waste, industrial wastewater, and industrial waste gas vary greatly in ERB implementation, and relatively few PMEs have implemented ERB. There is ample room for improving ERB implementation among these enterprises.

Besides, the mean and median of the PMEs under EEP regulation were not different. This means most enterprises differ slightly in the marketization level. But very few enterprises diverge significantly in that respect.

Furthermore, a large industrial concentration difference was observed between enterprises of different industries, suggesting that the sample enterprises engaged in fierce market competitions.

Concerning the form of ownership, the median stood at 1. Among the research samples, the domestic PMEs implement more ERB standardization than foreign-funded PMEs.

In addition, the PMEs did not have much difference in scale and surviving time, and all had a high equity concentration. Hence, the shareholders of each enterprise have a great say during ERB decision-making.

To disclose the influence of PMEs' ERB on its PB, this study carries out a regression analysis on variables like MI and ROA. The regression results in Table 2 show that the regression coefficient of PMEs' ERB on PB was smaller than zero, i.e., PMEs' ERB significantly suppresses PB. In other words, the PB of a PME will fall because of the implementation of ERB. This is probably because the economic benefit of production is delayed by only one cycle in our data analysis, while ERB benefit takes a long time to materialize, for PMEs need to pay an extra cost in implementing ERB. In addition, the asset-liability ratio has a significant negative correlation with PB. The generation of liability would drag down PB. Meanwhile, every other variable has a positive relationship with PB.

To make the above conclusion more reliable, a robustness test was performed on the policy-behavior-performance conceptual model. In the previous studies, the PMEs' ERB is mainly measured by the amount of environmental investment and its natural logarithm. This study modifies the measuring method of PMEs' ERB. According to the robustness test results in Table 3, EEP regulation still has a positive correlation with PMEs' ERB. This agrees with the empirical results in Table 2. The relationship between industry concentration and PMEs' ERB was approximately significant. It is confirmed that after the adjustment of the measuring method for PMEs' ERB, the variables still have significant correlations. Thus, our empirical model is highly robust.

Figure 3 shows the scatterplot of PMEs' ERB difference. It can be intuitively inferred that most PMEs' ERB standardization scores fell in the interval of [30, 60]. Therefore, although most PMEs in the region have implemented ERB rigorously, a few PMEs face a low standard level of ERB. These enterprises either invest very less to the innovation of green production processes or fall far short of the ideal ERB standard in terms of environmental investment and pollutant treatment level.

Finally, this study summarizes the ERB standard levels of PMEs in different industries (Figure 4). Ten industries were considered, including paper product manufacturing (T1), food processing and manufacturing (T2), wine and beverages manufacturing (T3), printing industry (T4), mineral product manufacturing (T5), furniture manufacturing (T6), pharmaceutical manufacturing (T7), metal processing (T8), electrical machinery (T9), and new energy power generation (T10). Among the PMEs in different industries, only those in T10 achieved a mean score above 50. The mean score of the PMEs in T1, T4, and T7 was below 30. The comparison between industries shows that the PMEs that are likely to pollute the environment do better in ERB control. The main reason is as follows: under the current EEP constraint, the traditional production and manufacturing industries receive more attention. These industries are forced to implement ERB well. In the same region, T1, T4, and T7 have not paid enough efforts to ERB implementation. More EEP guidance or mandatory constraint are needed.

## 5. Conclusions

This study explores the standardization of PME's ERB in the context of green economy. Specifically, the authors built a conceptual model for the action mechanism of the factors driving ERB standardization in enterprises, established an empirical model around the concept of policy-behavior-performance, and discussed the influence of PMEs' ERB over their PB. Drawing on the motivation-supervision theory, the authors also studied the influence of EEP supervision and motivation over the large panel PMEs' SSR and ERB. Through experiments, the authors obtained the descriptive statistics of the main variables in the empirical model based on the concept of policy-behavior-performance and conducted regression analysis and robustness test of two variables in the model, namely, MI and ROA. The results show that the proposed empirical model is highly robust. Then, the ERB difference between PMEs was displayed in the form of scatterplot, and the ERB standard levels of PMEs in different industries were summarized. Finally, it suggested providing more EEP guidance or mandatory constraint to the industries that have not paid enough efforts to ERB implementation.

In general, this research has several drawbacks. Model analysis and simulation analysis are the main tools in this research. These theoretical models and simulation systems help understand the basic laws of the objective world and the operation of objective phenomena. However, they are detached from the complex reality, failing to provide a perfect answer to real-world problems. To overcome the limitations, the future research will further explain the sample size, go deeper to the frontline of manufacturers, include the grassroots and ordinary people into the sample set, and survey green production more broadly. In addition, the hypothetical conditions of the theoretical model will be relaxed. The empirical research will be combined with qualitative and quantitative research, making the conclusions more scientific and reasonable.

## Figures and Tables

**Figure 1:** Conceptual model for the action mechanism of the factors driving ERB standardization in enterprises.

**Figure 2:** Driving mechanism of large panel PMEs' ERB.

**Figure 3:** Scatterplot of PMEs' ERB difference.

**Figure 4:** ERB standard levels of PMEs in different industries.

**Table 1:** Descriptive statistics of main variables.

Variable	ADU	MAR	FGT	HTQ	FEO	HR	CD	GV	TJ	EC	EQ	WE	MEU	DE
Quantity	241	265	239	284	215	269	236	294	251	238	229	205	273	282
Median	0.05	6.48	528.31	5	3	0.03	24.19	15	0.68	0.42	0.39	0.37	0.2	0.04
Mean	0.47	6.74	695.38	0.3	0.84	0.47	22.69	18.26	125	4.9	5.3	3.2	0.8	0.5
Standard deviation	0.07	2.58	648.75	0.7	0.49	1.7	1.36	4.58	8.6	1.5	5.4	0.7	2.6	1.7
Minimum	−1.3	−11.95	85.16	0.1	0.5	−9.6	22.48	5	12	0.7	0.2	2.4	0.1	0.9
Maximum	2.7	9.48	5216.36	1.6	1.8	4.3	23.48	25	5.37	8.6	4.18	6.2	1.02	7.4

**Table 2:** Regression results of PMEs' ERB on PB.

ZBL	HTQ	MEU	HR	ADU	CD	GV	TJ	EC	EQ	WE	MEU	DE
Ceef.	−0.847	0.032	0.015	−0.184	0.036	0.027	0.058	0.116	0.048	0.062	0.048	−0.169
StFn.	0.415	0.026	0.074	0.084	0.069	0.028	0.061	0.047	0.026	0.017	0.049	0.057
*T* value	−1.62	1.37	1.69	−2.47	1.39	1.25	3.95	3.48	2.37	1.84	0.69	−2.47
*P* value	0.058	0.196	0.268	0.015	0.169	0.192	0.025	0.013	0.028	0.047	0.369	0.042
95% confidence interval	−1.258	−0.015	−0.028	−0.169	−0.048	0.069	0.041	0.038	0.086	−0.025	−0.074	−0.359
	0.028	0.139	0.025	−0.036	0.027	0.039	0.052	0.258	0.069	0.042	0.196	−0.074
Sig	^*∗∗*^		^*∗∗∗*^			^*∗∗∗*^			^*∗∗*^			^*∗*^

^∗∗∗^ *p* < 0.01, ^∗∗^*p* < 0.05, ^∗^*p* < 0.1.

**Table 3:** Results of the robustness test.

ZBL	HTQ	MEU	HR	ADU	CD	GV	TJ	EC	EQ	WE	MEU	DE
Coef	−0.025	0.036	0.041	−0.084	0.049	0.062	0.038	0.139	0.042	0.036	0.046	−0.395
St.Err	0.015	0.062	0.041	0.053	0.018	0.069	0.042	0.069	0.084	0.029	0.037	0.018
*T* value	−2.25	1.36	0.84	−3.69	2.18	2.59	3.52	3.74	1.69	2.35	0.72	−3.95
*P* value	0.028	0.128	0.439	0.015	0.062	0.095	0.041	0.036	0.284	0.095	0.513	0.048
95% confidence interval	−0.015	−0.036	−0.048	−0.075	0.062	0.028	0.069	0.074	−0.073	0.095	−0.084	−0.462
	0.029	0.162	0.047	−0.039	0.014	0.095	0.062	0.162	0.048	0.026	0.139	−0.148
Sig	^*∗∗∗*^		^*∗∗*^		^*∗∗*^	^*∗*^			^*∗∗∗*^			^*∗∗*^

^∗∗∗^ *p* < 0.01, ^∗∗^*p* < 0.05, ^∗^*p* < 0.1.

## Data Availability

The data used to support the findings of this study are available from the corresponding author upon request.
